# Plumbagin Ameliorates Collagen-Induced Arthritis by Regulating Treg/Th17 Cell Imbalances and Suppressing Osteoclastogenesis

This article has been retracted.

**DOI:** 10.3389/fimmu.2018.03102

**Published:** 2019-01-08

**Authors:** Tingyu Wang, Han Qiao, Zanjing Zhai, Jun Zhang, Jinwen Tu, Xinyi Zheng, Niandong Qian, Hong Zhou, Eryi Lu, Tingting Tang

**Affiliations:** ^1^Department of Pharmacy, Shanghai Ninth People's Hospital, Shanghai JiaoTong University School of Medicine, Shanghai, China; ^2^Shanghai Key Laboratory of Orthopaedic Implants, Department of Orthopaedic Surgery, Shanghai Ninth People's Hospital, Shanghai Jiao Tong University School of Medicine, Shanghai, China; ^3^Department of Surgical Oncology, The University of Texas MD Anderson Cancer Center, Houston, TX, United States; ^4^Bone Research Program, ANZAC Research Institute, University of Sydney, Sydney, NSW, Australia; ^5^Department of Stomatology, Shanghai Renji Hospital, Shanghai JiaoTong University School of Medicine, Shanghai, China; ^6^Department of Orthopaedic Surgery, Shanghai Institute of Traumatology and Orthopaedics, Shanghai, China

**Keywords:** inflammation, plumbagin, arthritis, Th17 cells, osteoclast

## Abstract

**Objective:** Plumbago zeylanica L. (with plumbagin as its active ingredients) has been used for centuries to treat conditions such as joint swelling, fractures, and bacterial infections, suggesting that it possesses anti-inflammatory and immunosuppressive properties. In the present study, we evaluated the potential anti-arthritic activity and related mechanisms of plumbagin.

**Methods:** Collagen-induced arthritis (CIA) was initiated in Wistar rats with collagen type II. Plumbagin (2 and 6 mg/kg) was orally administered to rats with CIA from day 12 to day 32 post immunization. The effects of plumbagin on arthritis progression were assessed by paw swelling, clinical scoring, and histologic analysis. The percentage of Treg and Th17 were defined by flow cytometry or immunofluorescence (IF) staining. Bone erosion and resorption were assessed by micro-CT and histomorphometric analysis. Osteoclast differentiation was further determined by *in vitro* osteoclastogenesis assay. The molecular docking assay was used to determine the potential binding site of plumbagin.

**Results:** Treatment with plumbagin significantly inhibited arthritis development, as well as suppressed the local and systemic inflammation. Plumbagin reciprocally regulated pro-inflammatory Th17 cell and immunosuppressive Treg cell populations. In addition, plumbagin protected inflammation-induced bone loss by inhibiting osteoclast formation and activity. Plumbagin markedly suppressed RANKL-stimulated osteoclast-specific gene expression by repressing NF-κB signaling activation and MAP kinase phosphorylation. Further study via molecular docking assay demonstrated that plumbagin bound to MET169 of JNK kinase and LYS138 and SER183 of p38 kinase.

**Conclusion:** Plumbagin not only attenuates the immune-induced arthritis by inhibiting inflammation, but also protects bone erosion by directly inhibiting osteoclast formation and activity. These data suggest plumbagin is a promising new candidate drug for treating inflammatory joint diseases.

## Introduction

Rheumatoid arthritis (RA) is a systematic autoimmune polyarthritis that leads to joint swelling and deformity. Persistent inflammation in RA leads to synovial hyperplasia, articular cartilage degradation, and bone erosion (1).

Recent studies have found that Th17 and regulatory T cells (Tregs) play important roles in the pathogenesis of RA (2, 3). Th17 cells are pro-inflammatory T helper cells that play a dominant role in the production of the pro-inflammatory cytokines, such as interleukin-17 (IL-17), which serves as a marker of inflammation (4). Tregs, in contrast, are immunosuppressive cells that participate in the regulation of RA progression (5). In most cases, the balance between Th17 and Tregs characterized by low Th17/Treg ratio may be compromised in RA disease. The imbalance of Th17/Treg has been also reported in several inflammatory disorders, such as primary biliary cirrhosis and inflammatory bowel disease (6). In addition, Th17 cells may induce osteoclast formation and regulate bone resorption in RA by upregulating receptor activation of nuclear factor-κB ligand (RANKL) (7). Furthermore, IL-17 mediates bone resorption and proteoglycan loss, which cause joint degradation (8). Therefore, adjusting Th17 cell and Treg levels in RA patients enables us to control the inflammatory process and simultaneously inhibit osteoclastogenesis.

Plumbagin (5-hydroxy-2-methyl-1,4-naphthoquinone) is a small molecular weight compound derived from the roots of Plumbago zeylanica L, a traditional Chinese medicine (TCM). It has been used for centuries in China as an effective medicine to treat conditions such as joint swelling, fractures, and bacterial infections, suggesting that it possesses anti-inflammatory and immune-suppressive properties (9). There have been several recent studies focusing on the anti-cancer, anti-inflammatory, and immune-suppressive properties of plumbagin (10, 11). Our previous studies have shown that plumbagin inhibits the growth, invasion, and migration while induces the apoptosis of human breast cancer cells (12, 13). We also found that the combination of plumbagin and zoledronic acid (ZA) significantly and synergistically suppressed tumorigenesis (14, 15).

On top of all the above mentioned features, the anti-inflammatory properties of plumbagin are especially noteworthy and have been reported by various studies. In our previous study, we found that plumbagin effectively downregulated expression of pro-inflammatory mediators by inhibiting NF-κB and MAPK signaling in LPS-stimulated RAW 264.7 cells (16). Checker et al. reported that plumbagin has anti-inflammatory effects on lymphocytes (17, 18). Sheeja demonstrated that plumbagin can inhibit carrageenan-induced paw edema in rats by prolonging hotplate reaction time and shortening pain response durations in formalin-induced nociception (19). Luo suggested that plumbagin can effectively decrease the expression of the pro-inflammatory cytokines including interleukin 1 (IL-1), interleukin 6 (IL-6), and tumor necrosis factor alpha (TNF-α) and can also inhibit the phosphorylation of NF-κB in carrageenan-induced edema (20). In addition, Poosarla et al. reported that plumbagin has inhibitory effects on T cells (21). However, there have been no reports regarding the therapeutic effect of plumbagin on RA and the mechanism underlying the effects of plumbagin. Thus, in this study, we aimed to further evaluating the effects and the mechanisms of plumbagin on inflammation and inflammation-induced bone destruction in a rat RA model.

## Materials and Methods

### Collagen-Induced Arthritis Induction

Male Wistar rats (6–8 weeks old) were maintained for collagen-induced arthritis (CIA) modeling, as described previously (22, 23). Briefly, the rats were intradermally immunized on the backs of their tails with 100 μl of bovine collagen type II (CII, 2 mg/ml) in Incomplete Freund's adjuvant (IFA) on day 0, which was repeated on day 7 for booster immunization. To assess the influence of plumbagin (Sigma-Aldrich, St. Louis, MO, USA) on CIA, plumbagin (2 mg/kg in the low group and 6 mg/kg in the high group) was administered intra-gastrically to CIA rats from day 12 to day 32 after first CII immunization. CIA rats treated with PEG 2,000 served as vehicle group. Arthritis severity scores (expressed as the sum of the scores of the four limbs) and paw swelling (expressed as the average volume increase of the two hind paws) were assessed every other day by two independent observers (3). All animal experiments were performed in accordance with the guidelines of the Ethics Committee of Shanghai Ninth People's Hospital, Shanghai Jiao Tong University School of Medicine.

### Micro-CT and Histologic Examination

Rats were harvested on day 32 after the first CII immunization. The right hind limb of rats were dissected and fixed in 4% paraformaldehyde/PBS and analyzed by micro-CT using an Inveon Micro PET/CT system (Siemens Co., Knoxville, TN). Scanning was performed at 60 keV, 167 μA, and 1,475 ms without using a filter. In total, ~100 slices were collected at a resolution of 20 μm per pixel. The 3-dimensional (3D) structure and morphometry were reconstructed and analyzed in a double-blinded manner. Following micro-CT scan, the right hind limbs were fixed in 10% NB-formalin for 3 days and decalcified for 14 days in 14% EDTA and then paraffin-embedded. Three micrometer sections were cut and Alcian blue/H&E Orange G or TRAP staining were performed. For immunofluorescence (IF) staining, the sections were blocked with blocking solution (Thermo Scientific) and incubated with anti-RORγ (Novus Biologicals) or anti-Foxp3 (Santa Cruz Biotechnology) antibodies at 4°C overnight. The sections were then washed with PBS and incubated in the presence of Alexa fluorescence 594 or Alexa fluorescence 488 labeled secondary antibodies. The nucleus was visualized with DAPI (Vector Laboratories). All sections were analyzed by a Olympus BX43 fluorescence microscopy with cellSens Standard software.

### Cell Culture

Spleens were isolated from each group on day 32 after the first CII immunization, and minced in PBS to form cell suspensions. After lysing the red blood cells with 0.83% ammonium chloride, we filtered the splenocytes through a 70 μm cell strainer. The splenocytes were then incubated with FITC-conjugated CD4 monoclonal antibodies (mAb, Thermo Fisher Scientific Co., United States), and then sorted by FACSCalibur flow cytometry sorting (BD PharMingen), to obtain CD4+ T cells. Purified CD4+ T cells then incubated with or without plumbagin for 3 days under Th17 cell polarization conditions as described in the literature (3). Murine RAW264.7 cells (American Type Culture Collection, Rockville, MD, United States) and osteoblastic MC3T3-E1 and Kusao cells were cultured in α-MEM (Hyclone, Logan, UT, United States) containing 10% fetal bovine serum (FBS, Hyclone, Logan, UT, United States) and penicillin/streptomycin (Gibco-BRL, Gaithersburg, MD, United States). RANKL and M-CSF (Rocky Hill, NJ, United States) were added in the culture to induce osteoclast formation in RAW264.7 cells. MC3T3-E1 and Kusao cells incubated with or without plumbagin in osteogenic media were used to determine the effects of plumbagin on osteoblast activity.

### Flow Cytometry

The splenocytes were stimulated for 4 h with phorbol myristate acetate (PMA) and ionomycin (Sigma-Aldrich), as well as GolgiStop (BD Biosciences). Then the cells were surface labeled with FITC-conjugated CD4 mAb. After being permeabilized with Cytofix/Cytoperm solution (BD PharMingen), the cells were intracellularly stained with PE-Cy 5-conjugated Foxp3 or APC-conjugated IL-17 (R&D). All data were acquired and analyzed using the Accuri C6 (BD Biosciences) software included with the instrument.

### *In vitro* Alkaline Phosphatase (ALP) and Alizarin Red (ARS) Assay

To induce osteogenic differentiation, murine MC3T3-E1 and Kusao cells were cultured in osteogenic media (α-MEM supplemented with 10% FBS, 50 μg/ml ascorbic acid, 10 mM glycerophosphate, 100 nM dexamethasone, and 1% penicillin/streptomycin) with the indicated plumbagin concentrations. After the cells were incubated for 3 and 7 days, respectively, ALP staining was performed with the staining kit (Nanjing Jiancheng Chemical Industrial Co. Ltd., Nanjing, China), according to the manufacturer's instructions. After the cells were incubated for 21 days, ARS staining was conducted for 45 min at room temperature using 1% alizarin-red solution (pH 4.2; Sigma-Aldrich). Then, the cells were washed twice with deionized water until the orange color disappeared. ARS quantification was subsequently carried out using 10% cetylpyridinium chloride (Sigma-Aldrich) in 10 ml of sodium phosphate (pH 7.0; Sigma-Aldrich) to resolve the previous orange dye, and optical density (OD) values were measured at 620 nm with a microplate reader (Thermo Electron Corp., Waltham, MA, USA). These experiments were repeated independently for at least three times.

### Cell Viability Assay

Cell viability was measured using the Cell Counting Kit-8 (CCK-8) method. RAW264.7 cells were seeded in 96-well plates at a density of 8,000 cells/well and then treated with complete α-MEM containing M-CSF (30 ng/ml) for 24 h. After that, the RAW264.7 cells were treated with various plumbagin concentrations for an additional 24, 48, 72, or 96 h. Ten microliters of CCK-8 solution was added into each well at 37°C for 2 h, and OD values were determined with a microplate reader. IC_50_ (half maximal inhibitory concentration) values were also calculated after 48 h and 72 h. These experiments were repeated independently for at least three times.

### *In vitro* Osteoclastogenesis Assay

Murine osteoclast precursor RAW264.7 cells were treated with or without plumbagin at the indicated concentrations in complete α-MEM containing 30 ng/ml M-CSF and 50 ng/ml RANKL. The osteoclast differentiation medium was replaced every 2 days until mature multinucleated osteoclasts were formed, followed by tartrate-resistant acid phosphatase (TRAP) staining. TRAP-positive multinucleated cells containing at least three nuclei were classified as mature osteoclasts. These experiments were repeated independently for at least three times.

### ELISA

The left hind paws were harvested from each group and suspended in PBS. TNF-α and IL-1β levels in tissue homogenate supernatant as well as serum were measured with ELISA kits (Jiayuan Biotechnology, Inc. PRC; Boster Biotechnology Co., Ltd. PRC). IL-17 and TGF-β levels in the culture supernatants were also determined using ELISA kits (Neobioscience Technology Co., Ltd, PRC), according to the manufacturer's instructions.

### RNA Extraction and Real-Time PCR

RNA was extracted using TRIzol. Gene expression levels of RORγt, Foxp3, ACP5, ATP6V0D2, CTSK, DCSTAMP, and NFATc-1 induced by RANKL in RAW264.7 cells were measured via real-time PCR (ABI 7500, Applied Biosystems Inc., United States), according to the manufacturer's protocols. GAPDH was used as a quantitative control gene, and all reactions were run in triplicates. The sequences for the relevant primers were as follows: RORγt (F): 5′-CGCCTGGAGGACCTTCTACG-3′ and (R): 5′-ACAGCTCCATGAAGCCTGAG-3′; Foxp3 (F): 5′-TGAGCTGGCTGCAA TTCTGG-3′ and (R): 5′-ATCTAGCTGCTCTGCATGAGGTGA-3′; ACP5 (F): 5′-TC CTGGCTCAAAAAGCAGTTF-3′ and (R) 5′-ACATAGCCCACACCGTTCTC-3′; ATP6V0D2(F): 5′-GCCTCAGGGGAAGGCCAGATCG-3′ and (R): 5′-GGCCACCTCTTCACTCCGGAA-3′; CTSK (F): 5′-GGACCCATCTCTGTGTCCAT-3′ and (R): 5′-CCGAGCCAAGAGAGCATATC-3′; DCSTAMP (F): 5′-AAAACCCTTGG GCTGTTCTT-3′ and (R): 5′-AATCATGGACGACTCCTTGG-3′; NFATc-1 (F): 5′-GGGTCAGTGTGACCGAAGAT-3′ and (R): 5′-GGAAGTCAGAAGTGGG TGGA-3′; and GAPDH (F): 5′-TGGAGAAACCTGCCAAGTATGA-3′ and (R): 5′-CTCTCAGCTGTGGTGGTGAA-3′.

### Western Blotting

Murine osteoclast precursor RAW264.7 cells were pretreated with 5 μM plumbagin for 6 h, followed by stimulation with 50 ng/ml RANKL for 0, 5, 10, 20, 30, or 60 min. Cells were then lysed with RIPA buffer (Beyotime, Shanghai, China) for protein extraction. Equal volumes of protein lysates were resolved using SDS-PAGE and then transferred to polyvinylidene difluoride membranes (Millipore, Bedford, MA, United States). These membranes were incubated with the appropriate primary antibodies (Cell Signaling Technology, Danvers, MA, United States) at 4°C overnight before secondary antibody incubation (Abcam, Cambridge, United Kingdom) for 2 h at room temperature. The results were detected with an Odyssey V3.0 image scanner (Li-COR. Inc., Lincoln, NE, United States). The experiments were repeated independently for at least three times.

### Molecular Docking

Three-dimensional homology models of mouse JNK/p38 kinase domains were established with Modeler 9.12 using human JNK and p38 architecture as templates. The JNK/p38 stereo-chemical constructs were confirmed using PROCHECK. MolConverter and MarvinSketch were used to generate and refine the spatial coordinates of plumbagin, which was linked to the ATP docking pockets of JNK and p38 using the Lamarckian genetic algorithm based on AutoDock and AutoDock Vina. The resulting molecular model figures depicting binding activity were prepared using PyMOL visualization software.

### Statistical Analysis

All data are expressed as the mean ± SEM and were analyzed using Student's *t*-test (comparisons between two groups) or ANOVA followed by LSD and S-N-K test. *P* < 0.05 were considered statistically significant.

## Results

### Plumbagin Ameliorates the Progression of Inflammatory Arthritis

Paw swelling of all the rats were measured and scored every other day from day 12 until day 32 post type II collagen (Col-II) immunization. As shown in Figures 1A,B, arthritis developed in CIA rats treated with vehicle since day 12, which continued to increase and peaked approximately on days 24–26 after Col-II immunization. Low dose (2 mg/kg) and high dose (6 mg/kg) of plumbagin were orally administered to rats with CIA from day 12 to day 32. Compared with CIA rats treated with vehicle, plumbagin-treated CIA rats exhibited significantly attenuated arthritis, as determined by hind paw volume measurement, and arthritis scores (Figures 1A,B). The attenuated paw swelling in plumbagin-treated CIA rats was displayed by the representative images of the hind paws from rats of different groups taken on day 32 (Figure 1C).

**Figure 1:** Plumbagin (PL) treatment suppresses inflammatory arthritis in rats with collagen-induced arthritis (CIA). **(A,B)** Hind paw swelling measurement and time course of clinical arthritis in non-arthritic control rats (Ctrl), vehicle-treated CIA (CIA+Veh) rats, and CIA rats treated with low and high doses of plumbagin [CIA+PL(low) and CIA+PL(high)]. **(C)** Representative images of paw swelling. **(D,E)** Representative images of Alcian blue/H&E Orange G stained knee sections from different groups (original magnification ×50). Yellow arrowheads indicate sites of synovitis **(D)** and cartilage degradation **(E)**. **(F,G)** Protein levels of TNF-α and IL-1β in the supernatant of hind paw joint homogenate as measured by enzyme-linked immunosorbent assay (ELISA) on day 32. **(H,I)** Protein levels of TNF-α and IL-1β in rat plasma as measured by ELISA on day 32. Quantitative results are presented as mean ± SEM, and *n* = 10/group. ##*P* < 0.01 vs. non-arthritic control rats. ^*^P < 0.05; ^**^P < 0.01 vs. vehicle-treated CIA rats.

Compared to non-arthritic rats, histological examination of joints from CIA rats demonstrated severe synovial proliferation and inflammatory cell infiltration (Figure 1D), as well as cartilage destruction (Figure 1E). Plumbagin-treated CIA rats exhibited significantly alleviated inflammation and cartilage degradation when compared with the vehicle-treated CIA rats (Figures 1D,E). In consistence with the measurement and score of paw swelling, the supernatant of ankle joint tissue homogenate exhibited a down-regulation of the pro-inflammatory cytokines TNF-α and IL-1β in plumbagin-treated CIA rats when compared to CIA-vehicle rats (Figures 1F,G). In addition, there was also a systemic reduction of TNF-α and IL-1β levels resulted from plumbagin treatment as measured in plasma (Figures 1H,I). These results indicate that plumbagin inhibits joint inflammation, and suppresses pro-inflammatory cytokines both locally and systemically.

### Plumbagin Reciprocally Regulates Th17 Cells and Tregs *in vitro* and *in vivo*

Th17 cell/Treg imbalances play a pivotal role in RA pathology. To determine whether the Th17 and Treg cell populations were altered in plumbagin-treated CIA rats, the ratio of CD4^+^IL-17^+^ cells (Th17 cells) and CD4^+^Foxp3^+^ cells (Tregs) in the CD4^+^ T cells of spleen was assessed by flow cytometry. Compared to non-arthritic control rats, vehicle-treated CIA rats exhibited up-regulated CD4^+^IL-17^+^ cells which indicated increased Th17 cell population, as well as down-regulated CD4^+^Foxp3^+^ cells, which suggested decreased Treg cell population (Figures 2A–D). This Th17 cell/Treg imbalances associated with arthritis was rescued by plumbagin treatment. CIA rats treated with both low and high doses of plumbagin displayed decreased Th17 cell population and increased Treg cell population compared to vehicle-treated CIA rats (Figures 2A–D). Compared to non-arthritic control rats, the absolute number of Th17 cells was much higher and the absolute number of Treg cells was much lower in spleens of vehicle-treated CIA rats (Figures 2G,H). Plumbagin treatment significantly decreased the absolute numbers of Th17 cells and increased the absolute numbers of Treg cells in spleen of CIA rats (Figures 2G,H). In addition to cell population and absolute number evaluations, the gene expression levels of RORγt and Foxp3 as Th17 and Treg specific transcription factors were also measured in isolated splenocytes. In consistence with the flow cytometry results, RORγt mRNA levels were lower in plumbagin-treated CIA rats than in vehicle-treated CIA rats (Figure 2E). Conversely, Foxp3 mRNA levels were significantly higher in plumbagin-treated CIA rats than that in vehicle-treated CIA model in rats (Figure 2F). To examine whether plumbagin regulates Th17 cells and Tregs in inflamed joint, we performed immunofluorescence (IF) staining to measure RORγt and Foxp3 expression in the joint tissues from CIA rats treated with vehicle or plumbagin. As shown in Figures 2I–K, plumbagin treatment significantly decreased the numbers of Th17 cells and increased the number of Tregs in knee joint of CIA rats.

**Figure 2:** Plumbagin reciprocally regulates Th17 cells and Tregs in rats with CIA. **(A)** Representative flow cytometry profile of IL-17+ cell frequencies among CD4+ T cells in spleens collected from Ctrl, CIA+Veh, CIA+PL(low), and CIA+PL(high) rats on day 32. **(B)** Representative flow cytometry profile of Fopx3+ cell frequencies among CD4+ T cells in spleens collected from rats of different groups on day 32. **(C,D)** Quantitative analysis of IL-17+ and Fopx3+ cell populations in splenic CD4+ T cells from rats of different groups on day 32. **(G,H)** Th17 cells and Treg cells were counted in the spleens of different groups on day 32. **(E,F)** Gene expression of *ROR*γ*t* and *Foxp3* as assessed by qRT-PCR of splenocytes isolated from rats of different groups. **(I)** Immunofluorescence micrographs of RORγt (red) or Foxp3 (green) in the knee joint of the vehicle and plumbagin-treated CIA rats. DAPI (blue) was used to counterstain the nuclei. **(J,K)** Quantitative analysis of RORγt and Foxp3 cell numbers in joint tissues from CIA rats treated with vehicle or plumbagin (high dose). Quantitative results are presented as mean ± SEM, and *n* = 5/group. ##*P* < 0.01 vs. normal control rats. ^*^P < 0.05; ^**^P < 0.01 vs. vehicle-treated CIA rats.

To further confirm the regulatory effects of plumbagin on Th17 and Treg cell imbalances, we investigated the effects of plumbagin on Th17 cell differentiation and Foxp3 induction *in vitro*. CD4^+^ T cells from CIA rats were cultured under conditions favoring Th17 cell development with or without plumbagin. Consistent with *in vivo* results, *in vitro* treatment with plumbagin at the doses as low as 2.5 μM already significantly decreased Th17 cell population and increased Treg cell population (Figures 3A–D). Plumbagin treatments also resulted in decreased RORγt and increased Foxp3 mRNA expression in CD4^+^ T cells (Figures 3E,F). In addition, as the main cytokines mediating Th17 and Treg activities, respectively, the protein levels of IL-17 and TGF-β in the supernatants of CD4^+^ T cell cultures were measured by ELISA. The results demonstrated that plumbagin (2.5 to 7.5 μM) treatment decreased IL-17 levels and increased TGF-β levels under the conditions favoring Th17 cell development (Figures 3G,H).

**Figure 3:** Reciprocal effects of plumbagin treatment on Th 17 and Treg cell differentiation *in vitro*. Representative flow cytometry profile **(A,B)** and quantification **(C,D)** of IL-17+ and Fopx3+ cells in splenic CD4+ T cells isolated from CIA rats, which were cultured under Th17-polarizing conditions for 72 h with or without plumbagin in different concentrations. **(E,F)** Gene expression of *ROR*γ*t* and *Foxp3* as assessed by qRT-PCR of splenic CD4+ T cells isolated from CIA rats with different treatments. **(G,H)** Protein levels of IL-17 and TGF-β as measured by ELISA in the supernatants of CD4^+^ T cell cultures under different conditions. Quantitative results are presented as mean ± SEM, and *n* = 5/group. ^*^P < 0.05; ^**^P < 0.01 vs. vehicle-treated CIA rats.

### Plumbagin Attenuated Joint Bone Erosion and Proximal Tibial Bone Loss in CIA Rats

In addition to joint inflammation and cartilage degradation, the μCT analysis revealed significant severer bone erosions in the knee and hind paw joints of CIA-vehicle rats (Figure 4A, red arrowheads). In contrast, the bone erosions were mild in plumbagin-treated CIA rats. In order to detect whether plumbagin protected bone loss, we further determined changes in bone microarchitecture in the proximal tibiae. In comparison to non-arthritic rats, the tibial trabecular bone volume (%, BV/TV) was significantly reduced in CIA rats (Figure 4B). The reduction of trabecular bone mass in CIA animals was largely due to a reduction in trabecular thickness (Tb.Th, Figure 4C) and an increasing in trabecular separation (Tb.Sp, Figure 4D). In contrast, this trabecular bone reduction was effectively protected by plumbagin treatment as shown in Figures 4B–D. In addition to trabecular bone, tibial cortical bone volume, and thickness were also reduced in CIA rats. Again, this cortical bone loss was protected by plumbagin treatments (Figures 4E,F). Taken together, these data suggest that plumbagin exerts significant protective effects against bone destructions in CIA rats.

**Figure 4:** Plumbagin suppresses joint bone erosion and tibial bone loss in rats with CIA. **(A)** Representative reconstructed 3D micro-CT images of knee and hind paw joints of Ctrl, CIA+Veh, CIA+PL(low), and CIA+PL(high) rats to show joint bone erosion. Red arrowheads indicate sites of joint bone erosion. **(B–F)** Micro-CT parameters of trabecular bone mass and cortical bone mass are shown in **(B)**, trabecular bone volume (BV/TV), **(C)** trabecular thickness, **(D)** trabecular separation, **(E)** corticol bone volume, **(F)** corticol thinkness. **(G)** Representative histological images of tartrate-resistant acid phosphatase (TRAP) staining for osteoclasts (red) at a region distant to the site of inflammation in the proximal tibia of rats from different groups. Histomophometric quantification of **(H)** osteoclast number/bone surface (N.Oc/BS), and **(I)** osteoblast surface/bone surface (Ob.S/BS) in rats from different groups. Quantitative results are presented as mean ± SEM, and *n* = 5/group. #*P* < 0.05, ##*P* < 0.01 vs. normal control rats. ^*^P < 0.05; ^**^P < 0.01 vs. vehicle-treated CIA rats.

Joint destruction is caused by decreased bone formation and increased bone resorption, therefore, we examined whether plumbagin affected osteoblast and osteoclast activities that controls the balance of bone formation and resorption. Histomorphometric analysis revealed that osteoclast numbers were increased in CIA rats compared with non-arthritic normal rats, which was significantly reduced by plumbagin treatment (Figure 4G). In contrast, as shown in Figure 4H, CIA rats displayed the significantly decreased osteoblast surface compared to non-arthritic control rats, however, there was no significant difference of osteoblast surface between vehicle-treated CIA rats and plumbagin-treated CIA rats (Figure 4I). These findings suggest that plumbagin has protective effects on bone resorption in CIA rats, without affecting bone formation.

### Plumbagin Inhibits Bone Damage by Decreasing Osteoclast Formation

The effects of plumbagin on osteoblast differentiation were further evaluated in MC3T3 and Kusao cells. Figure 5A showed that osteogenic media significantly increased ALP activity in MC3T3 cells, with no apparent effects on ALP activity in Kusao cells after 3 days incubation. Plumbagin treatment at different concentrations (0.15–1.25 μM) did not affect ALP activity in either MC3T3 or Kusao cells after 3 or 7 days incubation (Figures 5A–C). ARS staining also confirmed that no significant effects on mineralized bone matrix formation in either MC3T3 or Kusao cells resulted from plumbagin treatment (Figures 5D,E). These data suggested that there was no significant effects of plumbagin on osteoblast activity.

**Figure 5:** Plumbagin inhibits osteoclastogenesis via suppressing osteoclast formation. **(A,B)** Representative images of ALP stained osteoblastic 3T3 and Kusao cells treated with or without plumbagin in different concentrations (0.15 −1.25 μM) for 3 and 7 days. **(C)** Quantitative analysis of 3T3 and Kusao cells positive for ALP staining. **(D)** Representative images of ARS stained osteoblastic 3T3 and Kusao cells treated with or without plumbagin in different concentrations (0.15–1.25 μM) for 21 days. **(E)** Quantitative analysis of 3T3 and Kusao cells positive for ARS staining. **(F)** Representative TRAP staining image of RAW264.7 cells under RANKL/M-CSF stimulation with or without plumbagin (1.25–5 μM). **(G,H)** Quantification of TRAP-positive multinucleated osteoclasts numbers and resorption areas. **(I,J)** Cell viability assessment of RAW264.7 cells treated with plumbagin (2.5–20 μM) for 48 h and 72 h. The IC50 values in RAW264.7 cells treated with plumbagin for 48 h and 72 h is 11.22 and 9.22 μM, respectively. Quantitative results are presented as mean ± SEM, and *n* = 5/group. ^*##*^, ^**^, ^&&^, *P* < 0.01 versus control in **(C)** and **(E)**. ^**^, *P* < 0.01 versus plumbagin 0 μM group in **(G)** and **(H)**.

To further determine the effect of plumbagin on bone resorption, *in vitro* osteoclast formation assay was performed. Plumbagin at 2.5 and 5 μM concentrations for 5 days significantly inhibited RANKL/M-CSF-induced osteoclast formation in RAW264.7 cells (Figure 5F). Quantification of TRAP-positive multinucleated osteoclasts numbers and areas confirmed a reduction of osteoclast activity resulted from plumbagin treatment as shown in Figures 5G,H. In addition, after 48 and 72 h incubation, plumbagin (0.25–1.25 μM) inhibited osteoclast formation in RAW264.7 cells, with IC_50_ values of 11.22 and 9.22 μM, respectively (Figures 5I,J). Taken together, these findings indicate that plumbagin significantly inhibits osteoclast formation with no effect on osteoblast differentiation.

### Plumbagin Suppresses Osteoclast Activity by Repressing NF-κB Signaling Activation and MAP Kinase Phosphorylation

Since plumbagin exerted inhibitory effect on osteoclast formation and activity, we further investigated the underlying mechanisms by examining the expression of osteoclast-specific genes. Figures 6A–E showed that plumbagin at the concentration of 1.25 and 2.5 μM (or 2.5 μM only) significantly inhibited the expression of *ACP5, ATP6V0D2, CTSK, DCSTAMP*, and *NFATc-1* induced by RANKL in RAW264.7 cells. Figure 6F showed that administration of RANKL stimulated pI-κBα and pP65 expression and decreased total I-κBα expression, which were significantly abrogated by the treatment of plumbagin (Figure 6F). Figure 6G showed that RANKL induced pERK, pJNK and pP38 expression levels without affecting t-ERK, t-JNK, and t-P38 expression levels. However, administration of plumbagin inhibited RANKL-induced pJNK and pP38 expression without affecting pERK expression, demonstrating that pJNK, and pP38 kinases are more likely to be the targets of plumbagin. This was further confirmed by the molecular docking assay, which demonstrated that plumbagin bound to MET169 of JNK kinase and LYS138 and SER183 of P38 kinase, providing potential inhibition sites at which plumbagin functioned against MAPK pathway (Figures 6H,I). Additionally, the expression levels of downstream c-Fos and NFATc-1, which are activated following JNK/P38 phosphorylation, were significantly inhibited by plumbagin (Figure 6J). These results indicate that plumbagin is able to target kinases and abrogate phosphorylation of these kinases, thereby decreasing expression levels of downstream functional proteins which are important in the development of arthritis.

**Figure 6:** Plumbagin downregulates RANKL-activated NF-κB and MAPK signaling during osteoclastogenesis. **(A–E)** Gene expression of osteoclast-specific genes (*ACP5, ATP6V0D2, CTSK, DCSTAMP*, and *NFATc-1*) as assessed by qRT-PCR of RAW264.7 cells under RANKL/M-CSF stimulation with or without plumbagin (1.25–5 μM) for 24 h. **(F)** Protein level of NF-κB signaling in RAW264.7 cells treated with RANKL and plumbagin for up to 60 min evaluated by Western blotting. **(G)** Protein level of MAPK signaling in RAW264.7 cells treated with RANKL and plumbagin for up to 60 min evaluated by Western blotting. **(H,I)** The potential binding sites of plumbagin against JNK and P38 kinase displayed by molecular docking assay. **(J)** Downstream osteoclastic protein (c-fos and NFATc-1) levels in RAW264.7 cells treated with RANKL and plumbagin for up to 5d evaluated by Western blotting. Quantitative results are presented as mean ± SEM, and *n* = 3/group.^**^P < 0.01 vs. plumbagin 0 μM group.

## Discussion

In the current study, we used the well-established CIA model to investigate effects of plumbagin on inflammation and inflammation-mediated bone damage in arthritis. Plumbagin significantly inhibited arthritis development by alleviating paw swelling and histological changes, as well as suppressing the joint tissue expression of TNF-α and IL-1β and their serum levels. This anti-inflammatory effects of plumbagin appeared through its reciprocally regulation of the populations of Th17, the inflammatory cell, and Treg, the immunosuppressive cells, indicating that plumbagin has the ability to reduce systemic and local inflammation. Plumbagin also protected inflammation-induced bone loss through its direct inhibition effects on osteoclast formation and activity via NF-κB pathway signaling activation and MAP kinase phosphorylation.

Th17 cells are a subgroup of CD4^+^ T cells that are capable of producing high levels of IL-17 and possess the specific transcription factor RAR-related orphan receptor gamma t (RORγt). In recent years, the role of Th17 in RA has been studied extensively. IL-17 levels are much higher in the synovial fluid of RA patients than in the synovial fluid of osteoarthritis patients (24). In RA synovial fibroblasts cultures, IL-17 induces the production of inflammatory cytokines (such as IL-6, IL-8, PGE2, and G-CSF) in a dose-dependent manner, and these effects can be blocked with the anti-IL-17 antibody (25). Blocking IL-17 using different methods including anti- IL-17 antibody, transgenic IL-17 knockout, transgenic *IL-17RA* knockout, and soluble IL-17 receptor protein alleviated arthritis in various models (26–29). On the other hand, both systemic and local (intra-articular) adenoviral IL-17 gene transfer exacerbated CIA (4).

CD4^+^CD25^+^ T regulatory cells (Tregs) possess the specific transcription factor Foxp3 and play pivotal roles in immunological tolerance and immune homeostasis. Treg levels and functions are decreased and impaired, respectively, in both RA patients and in CIA animal models (22, 23, 30, 31). In the present studies, Th17-Treg cell imbalance was observed in CIA rats with increased Th17 cell population and decreased Treg cell population, which was consistent with the clinic data of RA patients (30) Moreover, compared with non-arthritic control rats, the absolute number of Th17 cell was much higher and the absolute number of Treg cell was much lower in the spleen of vehicle-treated CIA rats. This imbalance was rescued by plumbagin, associated with decreasing RORγt mRNA levels and upregulating Foxp3 levels in the splenocytes of CIA rats, resulting in less server inflammation. Furthermore, plumbagin-mediated Foxp3 expression under Th17-polarizing conditions facilitated the conversion of Th17 cells to Tregs. The mechanisms of converting Th17 cells into Treg cells by plumbagin should be investigated in details in the future.

Bone erosion on the surface of inflammatory knee-joints and bone loss in proximal tibiae associated with joint inflammation were clearly demonstrated in CIA rats. Both micro-CT and histomorphometric analyses showed that plumbagin exerts protective effects against those CIA-related bone destruction. During RA progression, bone damage hinges on the balance between osteoblast and osteoclast cells. Our data strongly suggest that plumbagin exerts the direct effects on osteoclastogenesis through RANKL pathway. RANKL binds to RANK, expressed in the surface of osteoclast precursor cells, and then stimulates NF-κB and MAPK pathways (32) NF-κB activation begins with I-κBα phosphorylation, which increases downstream p65 translocation and phosphorylation, contributing to NF-κB signaling activation (33). In the RANKL-stimulated *in vitro* system, pretreatment of cells with plumbagin significantly decreased multinucleated osteoclast formation. In addition, plumbagin reduced RANKL-induced NF-κB p65 phosphorylation and I-κBα phosphorylation, suggesting that plumbagin influences NF-κB activation via these upstream effects. Plumbagin also affected MAPK pathway by attenuating JNK and p38 phosphorylation without impacting ERK phosphorylation. It was confirmed by molecular docking assay which revealed that plumbagin was able to target JNK and p38 kinase binding sites, thus inhibiting the subsequent phosphorylation and downstream activation of functional proteins, such as c-Fos and NFATc-1. The transcriptional factor NFATc1 is considered a trigger for osteoclast terminal differentiation, as NFATc1 deficient bone marrow macrophages cannot differentiate into multinucleated osteoclasts, even with RANKL stimulation (34). Upon activation, NFATc1 is translocated from the cytoplasm to the nucleus via a calcineurin-dependent mechanism and triggers the transcription of genes required for osteoclast differentiation, as well as bone resorption (34–36). Furthermore, it has been reported that NFATc1 directly binds to the ACP5, ATP6V0D2, CTSK, and DCSTAMP promoters. Interestingly, Western blotting and real-time PCR results in our study indicated that plumbagin decreases NFATc1 protein expression in osteoclasts through a transcription-dependent mechanism, resulting in the subsequent downregulation of *ACP5, ATP6V0D2, CTSK*, and *DCSTAMP* mRNA expression.

Of note, IL-17 have been shown to promoted osteoclast formation from CD14^+^ osteoclast precursor cells acquired from healthy donors by upregulating receptor activator of NF-κB (RANK) (8) Another study also reported that bone erosion and destruction in CIA is driven by Th17 cells by regulating RANKL-mediated osteoclast formation (7). In our study, plumbagin treatment significantly decreased the numbers of Th17 cells, and increased the number of Tregs in the inflamed joint of CIA rats. These indicated that the bone protection effects of plumbagin shown in the current study may be also resulted from its regulation of Th17 cells, however, more evidence is required in future investigations.

In conclusion, the findings of the current study have important implications regarding the potential application of plumbagin as a treatment of RA, as our data suggest that this therapy can not only alleviate inflammatory response which results in mitigating inflammation-associated bone destruction, but also protect bone loss directly.

## Author Contributions

All authors were involved in drafting the article or revising it critically for important intellectual content, and all authors approved the final version to be published. TW, EL, and TT designed the research. TW, HQ, and ZZ performed experiments and had full access to all of the data in the study. TW, HQ, ZZ, and JZ analyzed data. TW, HQ, XZ, NQ, EL, JT, HZ, and TT wrote the manuscript.

### Conflict of Interest Statement

The authors declare that the research was conducted in the absence of any commercial or financial relationships that could be construed as a potential conflict of interest.
